This article has been retracted.

# Efficacy of Dexamethasone versus Dexmedetomidine Combined with Local Anaesthetics in Brachial Plexus Block: A Meta-Analysis and Systematic Review

**DOI:** 10.1155/2022/7996754

**Published:** 2022-03-01

**Authors:** Ming Li, Pinghu Zhang, Duangao Wei

**Affiliations:** ^1^Department of Pharmacy, Affiliated Hospital of Yangzhou University, Northern Jiangsu People's Hospital, Yangzhou 225001, Jiangsu Province, China; ^2^Department of Pharmacy, Yangzhou University Medical College, Yangzhou 225009, Jiangsu Province, China; ^3^Department of Anesthesiology, Affiliated Hospital of Yangzhou University, Northern Jiangsu People's Hospital, Yangzhou 225001, Jiangsu province, China

## Abstract

**Background:**

Both dexamethasone and dexmedetomidine are commonly used local anaesthetic adjuvants in brachial plexus block to enhance the blocking effect. However, it is unclear which of the two drugs is more effective in a brachial plexus block. This article compares the effects of dexamethasone and dexmedetomidine combined with local anaesthetics in brachial plexus block through meta-analysis, availing information for current practice and future research.

**Methods:**

We conducted a search of the PubMed, Embase, Cochrane Library, and Web of Science databases to identify studies investigating the effects of dexamethasone and dexmedetomidine combined with local anaesthetics on brachial plexus block. The databases were searched from their inception to October 2021. Clinical randomized controlled trials were included. Two researchers independently conducted literature screening. The Cochrane System Review Manual was adopted for literature quality evaluation, whereas Stata 14.0 software aided in the meta-analysis. The duration of analgesia was the primary outcome indicator; whereas, the secondary outcome indicators included the duration of sensory block and motor block.

**Results:**

Seven articles were analysed, including 465 patients. Compared to the dexmedetomidine group, the dexamethasone group exhibited longer durations of analgesia (WMD = 111.29, 95% CI: 16.49–206.10, *P* = 0.021), sensory block (WMD = 173.20, 95% CI: 86.69–259.71, *P* < 0.0001), and motor block (WMD = 121.03, 95% CI: 12.87–229.20, *P* = 0.028).

**Conclusion:**

The present meta-analysis results affirm that dexamethasone is a better local anaesthetic adjuvant in brachial plexus block that enhances the blocking effect. Nevertheless, the existing heterogeneity warrants additional large-scale, multicentre, high-quality randomized controlled trials in the future for further verification and to provide more reliable clinical evidence.

## 1. Introduction

Compared to general anaesthesia, brachial plexus block has more merits, including low cost, fewer adverse reactions, less postoperative pain, and shorter hospital stay. It works both as an intraoperative and postoperative analgesia [1]. With advancements in ultrasound guidance technology, the application of brachial plexus block is crucial for the use of surgical anaesthesia in the upper limb. In contrast, a single brachial plexus block uses short-acting local anaesthetics, providing ineffective postoperative analgesia that impacts the patient's prognosis [2]. Postoperative pain rapidly increases the body's stress response. Consequently, the level of stress response substances in blood vessels increases, causing vasospasm. Neurohumoural factors stimulates the body's release of several damaging substances, such as catecholamines and prostaglandins, inducing strong contractions of the small blood vessels. Eventually, a vascular crisis occurs [3], which justifies why postoperative analgesia is particularly important.

Numerous reports have confirmed that dexamethasone and dexmedetomidine prolong the action time following the introduction of local anaesthesia to peripheral nerve block [4–7]. Combining dexamethasone or dexmedetomidine as a local anaesthetic adjuvant improves block characteristics, whether around the nerve or in the vein [8]. Multiple meta-analyses have convincingly demonstrated its effectiveness in prolonging the duration of brachial plexus block pain relief [9–12]. Most published trials of dexamethasone and dexmedetomidine have compared these adjuncts to the control, with very few one-to-one comparisons [13]. Although some scholars have conducted indirect meta-analyses on the auxiliary effect of dexamethasone versus dexmedetomidine in brachial plexus blocks [13], there is no report on the direct comparison of dexmedetomidine combined with local anaesthetics in brachial plexus blocks. Thus, no substantial evidence has implicated dexamethasone as a better adjuvant.

Recently, research on the direct comparison of dexmedetomidine combined with local anaesthetics for brachial plexus block is increasing. There is an urgent need to update the meta-analysis of dexamethasone combined with local anaesthetics directly comparing dexmedetomidine combined with local anaesthetics for brachial plexus block to determine whether dexamethasone is a better adjuvant and to provide supporting evidence for clinical decision-making.

## 2. Methods

This review was conducted in accordance with the Preferred Reporting Items for Systematic Reviews and Meta-Analyses guidelines (PRISMA). The review protocol was registered on the Open Science Framework (registration number: DOI 10.17605/OSF.IO/NQ5XM).

### 2.1. Literature Search

Computer searches in PubMed, Embase, Cochrane Library, and Web of Science were performed. The search terms included “dexamethasone,” “dexmedetomidine,” “brachial plexus block,” “nerve block,” “perineural”, and “intravenous.” The databases were searched from their inception to October 2021.

### 2.2. Selection Criteria

Inclusion criteria included randomized controlled trials of brachial plexus block, adult patients aged 18 years and older, and a group of local anaesthetics combined with dexmedetomidine or local anaesthetics combined with intravenous dexmedetomidine and another group of local anaesthetics combined with perineuronal dexamethasone or local anaesthetics combined with intravenous dexamethasone. Exclusion criteria included reviews, animal experiments, case reports, and meta-analyses.

### 2.3. Data Extraction

Two researchers screened the retrieved documents independently. After preliminary browsing based on the title and abstract, duplicate documents were deleted. Documents that did not meet the inclusion criteria were excluded. The full texts of the documents likely to be included were downloaded and read carefully. In case of inconsistent opinions, two researchers reevaluated the quality of the full text and engaged in discussion to reach a consensus. In any case that there was no agreement, a third researcher decided on whether to include the literature. We extracted the following patient characteristic data: main author, year of publication, country, type of surgery, sample size, nerve block approach, operative site, neurolocation technology, drug type, and dose.

### 2.4. Literature Quality Evaluation

Two researchers evaluated the retrieved literature independently using the Cochrane Systematic Review Manual's bias risk assessment tool for randomized controlled trials. The tool incorporated the following questions: whether the random sequence was accurately generated, whether the allocation concealment was correct and sufficient, whether the blind method was applied, whether the ending data were complete, and whether there was any loss. Each risk of bias was classified into low risk, high risk, or unclear.

### 2.5. Outcomes

The primary outcome measure was the duration of analgesia, defined as the time interval between the completed injection of local anaesthetics and the first administration of analgesics. The secondary outcome indicators included the duration of sensory block and duration of motor block, defined as the time interval between the completion of the local anaesthetic injection and recovery of the nerve block.

### 2.6. Statistical Analysis

Meta-analysis was performed using Stata 14.0 (Stata Corp, College Station, TX, USA). The duration of analgesia, sensory block, and motor block were considered continuous variables, expressed as weighted mean difference (WMD) and 95% confidence interval (95% CI). The heterogeneity across the results of the included studies was analysed using the *χ*^2^ test (test level is *α* = 0.1). *I*^*2*^ was applied to quantitatively determine the size of the heterogeneity. Notably, at *P* *>* *0*.1 and *I*^*2*^<50%, the data were considered nonheterogeneous, and the fixed effects model was adopted; however, at *P* < 0.1 and *I*^*2*^>50%, the data were considered heterogeneous, and the random-effects model was adopted. Next, the causes of heterogeneity were analysed. This was followed by subgroup and sensitivity analyses of the possible causes of heterogeneity. A funnel chart was generated to evaluate possible publication bias and small sample bias using Egger's test and Begg's test. *P* < 0.05 denoted significant differences.

## 3. Results

### 3.1. Literature Retrieval Results

A total of 396 articles were retrieved from the preliminary search. After screening, 7 articles [14–20] were finally included for analysis, with 465 patients. The literature screening process is shown in Figure 1.

### 3.2. Basic Characteristics of Literature

The 7 trials [14–20] were published from 2014 to 2020 and distributed as follows: India had 4 trials [14, 16, 18, 19], Iran had 1 trial [20], Korea had 1 trial [17], and Chile had 1 trial [15]. The nerve block approach included interscalene groove, axillary approach, infraclavicular block, and supraclavicular approach. A type of forearm surgery was performed. Neural localization techniques involved ultrasound, nerve stimulation, and ultrasound combined with nerve stimulation. The basic characteristics of the literature are given in Table 1.

### 3.3. Risk of Bias Assessment

The randomization and allocation methods in one study [15] were unclear. The remaining studies showed low-risk bias. The quality evaluation results of the included literature are shown in Figure 2.

### 3.4. Meta-Analysis Results

#### 3.4.1. Duration of Analgesia

A total of 5 studies [15, 16, 18–20] reported the duration of analgesia. Based on a random-effects model, the heterogeneity results were *I*^*2*^ = 97%, *P* *<* 0.001. Compared to the dexmedetomidine group, the dexamethasone group prolonged the duration of analgesia (WMD = 111.29, 95% CI: 16.49–206.10, *P* = 0.021) (Figure 3). The *I*^*2*^ value and effect scale did not change significantly after the sensitivity analysis via the article-by-article elimination method, demonstrating that the research results were robust (Figure 4).

#### 3.4.2. Duration of Sensory Block

The duration of sensory block was reported by 7 studies [14–20]. The heterogeneity result was *I*^*2*^ = 93.5%, *P* *<* 0.001, based on the random-effects model. Compared to the dexmedetomidine group, the dexamethasone group had a prolonged sensory block duration (WMD = 173.20, 95% CI: 86.69–259.71, *P* < 0.0001) (Figure 5). There was no significant change in the *I*^*2*^ value or effect scale after the sensitivity analysis via the article-by-article elimination method, demonstrating that the research results were robust (Figure 6).

#### 3.4.3. Duration of Motor Block

The duration of motor block was reported by 6 studies [14–16, 18–20]. The heterogeneity result was *I*^*2*^ = 96.7%, *P* *<* 0.001, based on the random-effects model. Compared to the dexmedetomidine group, the dexamethasone group prolonged the duration of motor block (WMD = 121.03, 95% CI: 12.87–229.20, *P* = 0.028) (Figure 7). There was no significant change in the *I*^2^ value after the sensitivity analysis via the article-by-article elimination method. When we excluded articles by Adinarayanan et al. 2019 [14], Aliste et al. 2019 [15], Kumar 2014 [16], and Verma 2016 [19], the result was reversed. From this, we proved that the research results were not robust and thus needed further verification (Figure 8).

#### 3.4.4. Publication Bias

We applied Egger's test and Begg's test to evaluate publication bias. The duration of analgesia, sensory block, and motor block all had no publication bias (Begg's *P* = 0.624, Egger's *P* = 0.549; Begg's *P* = 0.881, Egger's *P* = 0.852; Begg's *P* = 0.573, Egger's *P* = 0.573) (Figures 9–11).

## 4. Discussion

For the first time, this meta-analysis directly compared the effects of dexamethasone versus dexmedetomidine as an adjuvant for local anaesthetics on brachial plexus block. Of note, compared to dexmedetomidine, dexamethasone combined with local anaesthetics significantly prolonged the duration of brachial plexus block analgesia, sensory block, and motor block.

A previous network meta-analysis by Albrecht et al. [13] implicated both dexamethasone and dexmedetomidine as effective adjuvants for brachial plexus block, and they also prolonged the sensory/motor block time. Of note, dexamethasone may be a better adjuvant, as it is associated with a longer duration of analgesia than dexmedetomidine but does not extend the sensory/motor block time. However, this evidence is of low quality. A direct comparison between dexamethasone and dexmedetomidine has yet to be published. With this, we conducted an updated systematic review of the current problems and collected RCTs from 2014 to 2020 for quantitative analysis. Indeed, the conclusion that dexamethasone combined with local anaesthetics prolongs the effect of brachial plexus block was validated.

At present, dexamethasone is commonly used in brachial plexus nerve block regardless of the perineural or intravenous route [21–24]. The analgesic mechanism of dexamethasone has the following aspects. (1) It potentially plays a major role by inhibiting the reduction of peripheral phospholipase, cyclooxygenase, and lipoxygenase. This is supported by the finding that the degree of prolonged blockade has the same hierarchical order as the anti-inflammatory ability of glucocorticoids and is completely reversible following the administration of specific glucocorticoid receptor antagonists [25]. (2) Dexamethasone reduces the production of bradykinin, which increases the pain of inflamed tissues and surgical areas. (3) Decreasing the concentration of neuroprotein secreted by the peripheral nervous system also plays a part in improving the analgesic effect. (4) Local effects include blocking the transmission of nociceptive unmyelinated C fibres and inhibiting the discharge of ectopic neurons [26]; this effect may be generated by changing the function of potassium channels in excitable cells.

In another retrospective analysis, Cho et al. [12] added dexamethasone to local anaesthetics for brachial plexus block. The results showed that dexamethasone extended the analgesic time of long-acting local anaesthetics from 730 min to 1306 min, with an average extension of 576 min; extended the analgesic time of intermediate-acting local anaesthetics from 168 min to 343 min, with an average extension of 175 min; and extended the motor block time from 664 min to 1102 min. Albrecht et al. [27] found in their systematic review of the safety and effectiveness of dexamethasone combined with local anaesthetics for peripheral nerve block that dexamethasone combined with short-acting or intermediate-acting local anaesthetics could prolong the analgesia time by an average of 233 min. Collectively, anaesthesia can prolong the analgesia time by an average of 488 min. Increasing the local dose of dexamethasone from 4 mg to 10 mg implies that the block time is not significantly prolonged; whereas, intravenous medication and peripheral medication exert similar effects. Furthermore, a meta-analysis by Huynh et al. [28] demonstrated that compared to when local anaesthetics were used alone, the addition of 4–8 mg of dexamethasone to the authorities' anaesthetics significantly shortened the onset time of sensory and motor block by approximately 1 min. Additionally, the analgesic time and motor block time were extended by an average of 351 min and 277 min, respectively. The latest research shows that compared with placebo, the perineural or systemic use of dexamethasone equally extends the block time [8].

This study has a few limitations. The meta-analysis results of the duration of analgesia, sensory block, and motor block are highly heterogeneous. Since we included only 7 articles, the information provided was limited. The subgroup analysis could not be performed based on the dose of dexamethasone and nerve block approach. Perineural administration of 4.0–5.0 mg dexamethasone has shown to provide a longer duration of sensorimotor block and analgesia than intravenous injection [7, 29]. However, we cannot rule out that a higher dose of dexamethasone can selectively support the intravenous injection route to achieve a potentially equivalent effect to that of peripheral administration. However, Sehmbi et al. [8] in their network meta-analysis of different routes of administration showed that the quality of evidence for the use of perineural and intravenous routes to administer dexamethasone was low and extremely low. In addition, it is elusive whether different blocking approaches can provide different results. Last, after sensitivity analysis, the source of heterogeneity was not revealed; this may be related to the type, concentration, volume of local anaesthetics, adrenaline, and race. These factors must be explored in future research.

## 5. Conclusion

The present study demonstrates that dexamethasone combined with local anaesthetics can significantly extend the time of brachial plexus block. However, owing to the high heterogeneity in the findings, additional large-scale, multicentre, high-quality randomized controlled trials are warranted for further verification to obtain more reliable clinical evidence.

## Figures and Tables

**Figure 1:** Flow diagram of the literature search strategy.

**Figure 2:** Authors' judgements regarding risk of bias for included studies.

**Figure 3:** Forest plot demonstrating duration of analgesia.

**Figure 4:** Sensitivity analysis for duration of analgesia.

**Figure 5:** Forest plot demonstrating duration of sensory block.

**Figure 6:** Sensitivity analysis for duration of sensory block.

**Figure 7:** Forest plot demonstrating duration of motor block.

**Figure 8:** Sensitivity analysis for duration of motor block.

**Figure 9:** Begg's funnel plot of duration of analgesia.

**Figure 10:** Begg's funnel plot of duration of sensory block.

**Figure 11:** Begg's funnel plot of duration of motor block.

**Table 1:** Trial characteristics.

Author, year	Country	Sample size		Nerve block approach	Operative site	Technique	Type, concentration, and volume of local anaesthetics	Concentration and volume of dexamethasone	Concentration and volume of dexmedetomidine
		Dexamethasone	Dexmedetomidine						
Yaghoobi, 2019	Iran	25	26	Infraclavicular block	Forearm surgery	Ultrasound	Lidocaine 2%, 28 ml	2 mL (8 mg)	2 mL (1 *µ*g/kg)
Verma, 2016	India	50	50	Interscalene groove	Forearm surgery	Nerve stimulation	Ropivacaine 0.5%, 30 ml	2 mL (8 mg)	1ml (50 *µ*g)
Singh, 2020	India	20	20	Supraclavicular approach	Forearm surgery	Ultrasound	Ropivacaine 0.5%, 30 ml	3 mL (8 mg)	2 mL (1 *µ*g/kg)
Lee, 2016	Korea	17	17	Axillary approach	Forearm surgery	Ultrasound + nerve stimulation	Ropivacaine 0.5%, 20 ml	2 mL (10 mg)	2 ml (100 *µ*g)
Kumar, 2014	India	30	30	Interscalene groove	Forearm surgery	Ultrasound + nerve stimulation	Bupivacaine 0.25%, 40 ml	2 mL (8 mg)	2 mL (50 *µ*g)
Aliste, 2019	Chile	60	60	Infraclavicular block	Forearm surgery	Ultrasound	35 mL of lidocaine 1% bupivacaine 0.25% with epinephrine 5 g/ml	5 mg	(100 *µ*g)
Adinarayanan, 2019	India	30	30	Supraclavicular approach	Forearm surgery	Ultrasound + nerve stimulation	Bupivacaine 0.5%, 25 ml	2 mL (8 mg)	2 mL (1 *µ*g/kg)

## Data Availability

The data used to support the findings of this study are available from the corresponding author upon request.
